# Biomechanical Simulation of Peyronie's Disease

**DOI:** 10.1155/2021/6669822

**Published:** 2021-03-13

**Authors:** Pavel Drlík, Vladimír Červenka, Jan Červenka

**Affiliations:** ^1^Central Military Hospital in Prague, Czech Republic; ^2^Cervenka Consulting s.r.o., Prague, Czech Republic

## Abstract

A pathological disorder of human penile function, known as Peyronie's disease, is characterized by the formation of plaque particles within the tunica albuginea. The plagues in the shape of rigid plate form in the scars as a result of the imperfect healing process. Due to high stiffness, plagues are the source of pain and anomalous deformations during erectile penis function. The authors simulate the biomechanical behavior of the penile structure by a 3D finite element model. The numerical model is based on the real geometrical shape and the tissue structure with consideration of large nonlinear deformations. The penile erection is modeled by the initial strains imposed on the corpus cavernosa. The stress analysis is performed in a case study of various plague locations. The Peyronie's syndrome manifested by the penis angular deviation simulated by the analysis is compared with the clinical data. The computational simulations provide a rational explanation for the clinical observations on patients. The objective is to apply the proposed modeling approach for the development and validation of treatment methods based on the application of shock waves.

## 1. Introduction

Peyronie's disease is characterized by a fibrous rigid scar (plaque) or indurated area in the tunica albuginea causing penile pain and penile curvature during erection, reducing the possibility of intercourse. Physical manifestation includes penile curvature, hinging, narrowing, shortening, and painful erections. Attempts to explain the pathogenesis and etiology of this frustrating disease are dated from the 13th century. This disease was named after François de la Peyronie [1], who worked on the study of induratio penis plastica, and recommended therapeutic approaches in the treatment of this disease. The etiology of this disease is currently not completely understood. Only a few studies have high merit of credibility, and the remaining studies had a low level of evidence.

The recent advances in biomechanics offer a rational scientific approach to its treatment by the mechanical modeling of the erectile process based on the structural analysis. Gefen et al. [2] and Gefen et al. [3] developed a computational model and investigated the stress states of the penis with Peyronie's plague. Their model was a 2D representation, in which the stress analysis of the penis cross-section was considered. In this model, the tunica albuginea was the only ligament forming the resisting structure. The corpus cavernosa was not represented by solid elements but substituted by the internal pressure acting inside on the tunica albuginea. Timm et al. [4] used a model based on 3D geometry and the internal pressure in the corpus cavernosa with the aim to simulate the buckling strength of the penis (stability limit). The mechanics of the Peyronie's disease and the effect of the fibrotic plague have not been extensively studied by 3D models.

The authors of this paper have investigated the question of the effect of a rigid plague on the behavior of the soft tissue structure of the penis. They have developed a 3D structural model reflecting the real penile structure. The penile anatomy is quite complex in detail, but only some of its constituents are relevant for the problem of the Peyronie's disease investigated here. The cross-section of the penis in the computational model is shown in Figure 1. It includes the corpus cavernosa as a driving agent of the erection and the tunica albuginea as a resisting ligament. The skin is just a cover layer with a negligible structural effect, and the glans tissue is needed to provide a pressure closure of the corpus cavernosa. Remaining components of the penis anatomy, such as corpus spongiosum, urethra, artery, veins, and nerves, are omitted in the numerical model since due to a low tissue stiffness they are not significant for the penis mechanical response.

In the computational model, the erectile function demarcated by the penis deformation is driven by the volume expansion of the corpus cavernosa, considered as a loading effect by the imposed initial strain. This approach is different from the other approaches described in the literature ([2, 3], Timm et al. 2008 [4]). It represents a robust approach and allows to control the deformation behavior of the model reflecting a real behavior. The numerical simulation was made using the commercial software ATENA (Cervenka et al. [5]).

## 2. Computational Model

The finite element model of the penis is illustrated in Figure 2. The penis length in the placid state is assumed to be 68 mm. The external dimensions of the cross-section are 23.6 × 17.5 mm (width × thickness). The size of each corpus cavernosa is 9 × 11.7 mm, the thickness of the tunica albuginea is 1.2 mm, and the skin on the sides is 1 mm. The dimensions are chosen to correspond on average to the real conditions of the penis anatomy.

The finite elements used for the penis body are the quadratic isoparametric brick elements with 20 nodes. For the glans, quadratic tetrahedral elements with 10 nodes (each node is with 3 DOF) were used. These high-order elements assume a linear strain distribution within the element, which enables a relatively accurate simulation of real stress and strain states. In the case of the elastic material, it means a linear stress distribution within the element. The updated Lagrangian approach is used for the modelling of this geometrically highly nonlinear problem. This means that all coordinates are updated, and all mechanical tensors are assembled at time *t*. The finite element simulation system ATENA [5] that was used throughout this study is based on the following governing equations in the weak form over the domain *V* for the time interval Δ*t* and iteration (*i*) in the nonlinear iterative process:

(1) ∫tVStt+Δtiji ∂εtt+ΔtijitdV=t+ΔtR,

where *S*_*ij*_^(*i*)^ is the 2nd Piola-Kirchoff stress tensor and *ε*_*ij*_^(*i*)^ is the Green Lagrange strain tensor at iteration *i* which take the following forms:

(2) Stt+Δtiji=ρtρt+Δt  xt+Δtti,mi  t+Δtτmni  xt+Δttj,ni,

(3) εtt+Δtiji=12utt+Δti,ji+utt+Δtj,ii+utt+Δtk,ii utt+Δtk,ji,

where ^*t*^*ρ*/^*t*+Δ*t*^*ρ* is a ratio of material density at the time *t* and *t* + Δ*t*, ^*t*^*ρ*=^*t*+Δ*t*^*ρ* det(_*t*_^*t*+Δ*t*^*F*_*ij*_); _*t*_^*t*+Δ*t*^*F*_*ij*_ = _*t*_^*t*+Δ*t*^*x*_*i*,*j*_ is the deformation gradient tensor to a position at the time *t*; ^*t*+Δ*t*^*τ*_*mn*_ is the Cauchy stress tensor at the time *t* + Δ*t*; _*t*_^*t*+Δ*t*^*x*_*i*,*m*_ is the derivative of point coordinates at the time *t* + Δ*t* to the configuration at the time *t*; and _*t*_^*t*+Δ*t*^*u*_*i*_=^*t*+Δ*t*^*x*_*i*_−^*t*^*x*_*i*_ is the *i*-th element of a vector of displacement increments at the time *t* + Δ*t*.

_*t*_^*t* + Δ*t*^ *R* represents the virtual work of the external forces at the time *t* + Δ*t*. This formulation assumes incremental loading in time intervals Δ*t*. The energetic conjugate quantities of 2nd Piola-Kirchhof and Green-Lagrange strain tensors enable to simulate load increments with large translations and rotations.

The boundary conditions are applied as displacement constraints fixed on the penile base surface in the axial direction *Z*. Besides, spring supports representing the reaction of the abdominal structure were applied on the base surface in *X* and *Y* directions, at 1 N/mm^3^.

The loading is applied through imposing the initial strain on the volume of the corpus cavernosa (Figure 2) by the value 0.7 in the axial direction *Z* and 0.4 in radial directions *X* and *Y*.

The choice of the material model is the result of a research study in which existing data from the literature were considered. In the first attempt, the corpus cavernosa was modeled as a soft material with internal pressure due to the blood represented by the initial stress. The model was similar to Gefen et al. [2] and Timm et al. [4] in which the tunica albigunea is inflated by the blood pressure from the corpus cavernosa. However, such a model does not properly reflect the mechanical action of the corpus cavernosa, namely, a penis deviation due to plague. Therefore, an alternative approach was chosen, in which the erectile action is simulated by the imposed strains on the corpus cavernosa body. This allows modeling a penis bending but requires sufficient stiffness of the corpus cavernosa body. The linear elastic material was chosen for all components of the penis structure with the geometrically nonlinear formulation of Green-Lagrange strains (3) to accommodate large deformations. A linear elastic material is assumed in this study for all materials. The parameters of the plague are according to Mente and Lewis [6]. The elastic modulus for the tunica albuginea was experimentally determined by Bitsch et al. [7] to be about 12 MPa. The list of material parameters used in the study is shown in Table 1. The material properties of the glans are not significant in this analysis, and elastic modulus was assumed to be 10 MPa and Poisson's ratio 0.4. The elastic properties for the corpus cavernosa are relatively high mainly due to the adopted initial strain approach, which requires a higher stiffness value to recover the expected behavior. These properties should correspond to the average properties of the corpus cavernosa in the state of erection and do not consider its detailed complex fibrous-fluid microstructure.

## 3. Case Study

This computational study is aimed at simulating the effect of plagues located within the tunica albuginea. The plaque size was 5 × 20 mm (tangentially × axially) and partially occupied the ligament volume. It was positioned at a distance of 10 mm from the penis base. The variety of plague positions in the radial orientation is indicated in Figure 3. Case 0 is without plague and serves as a reference to healthy conditions. Case A with two plagues is a frequently observed clinical case. Cases B to D are representing different plague locations.

Figure 4 shows the simulation of the penile deformations of all studied cases in the real scale 1 : 1. Deformations are accompanied by the stress fields and can be described by Von Mises stresses, typically used for the assessment of the material failure. By comparing Figure 5 (Case 0 normal) and Figure 6 (Case A with plague), a plague effect on the stress distribution can be observed. In the normal condition, the stress field is quite uniform on average 10 MPa. In contrast, with a plague, the stress field is irregular with maxima up to 30 MPa in concentrations, indicating an increase by factor 3 within the tunica albuginea. In the plague, the stress reaches the values of more than 50 MPa, indicating a stress intensity increase factor of about 5.

For brevity, a presentation of the detailed results of all cases is not shown. However, a summary of the results is given in Table 2, from which general conclusions can be drawn. The consequences of plague extent and location on the pathologic deformations are quite evident. The penile deviation from the normal state is in the radial direction of the plague location. The more extensive plague size produces a larger deviation and a shorter penis elongation.

## 4. Confirmation by Clinical Investigation

The first author performed an investigation of the Peyronie's symptoms, Drlik [8], within the research of treatment by the shock waves. The measurement of penis angular deviation due to Peyronie's disorder was performed on a group of 125 patients. The result of the clinical study is illustrated by the histogram of penile deviations shown in Figure 7. The range of deviation was from 5 to 90 degrees with the mean value at 49.6 degrees and the coefficient of variation 0.42 indicating a rather high random variability. Simulation Case A corresponds to the average of the clinical data. The results of the simulations are depicted by red marks. In general, the experimental data confirm the mechanical behavior documented in this study. Of course, due to the reduced extent of the numerical study limited to four cases, a wide range of clinical behavior was not covered. The significant variability of deviations observed in the clinical investigation can be attributed to a large variability of the parameters, namely, the plague size and location, and material properties of tissues. Furthermore, the present study does not include a disease stage with the plague extending into the corpus cavernosa, which could further increase the scatter of the results.

## 5. Clinical Application

Although a conservative therapy, which includes an application of Xiapex (clostridial collagenase) and shock pulses applied to the scar plagues, developed by the author, is relatively highly successful (in about 70-75% of patients), for a certain group of patients, an improvement is not observed, and a surgery is offered. The surgeries are aimed at the adjustment of penis angulation and at the restoring of a satisfactory sexual intercourse. It is always necessary to discuss with the patients the course of surgery and potential risks involved. The specific problems associated with this therapy are penis shortening, erectile and sensitivity malfunctions, recurrence of angulation, palpable stitches, and often a necessity to perform a circumcision within the surgery. Serious complications can arise due to inflammatory states and a development of cavernous scars in the erectile bodies. This can lead to serious malfunctions and an inability of satisfactory intercourse.

In this therapy, two classes of surgical methods are recognized. In the first method, referred as “shortening,” a resection is applied to the concave side of penis. In the second method, referred as “lengthening,” a plague scar is resected and replaced by a patch gained from the patient's own muscle. An example of the later method performed by the first author in a surgical procedure is illustrated in Figures 8 and 9.  Figure 8 shows the deformed penis under the artificial erection before a surgical correction, which confirmed the simulated predictions shown in Figure 4.  Figure 9 shows a state after resection before a patch implantation.

Based on our experience, a 3D model of penis anatomy is very supportive and helpful in planning a surgery of the specific patient. A mechanical model of penis angular deformation during the erection and its detail shape and direction provides a virtual simulation platform for the planning of surgery and enables to choose optimal parameters and predict the resulting effects. It supports the important decisions to be made in the planning phase of the therapy.

## 6. Concluding Remarks

The plague occurrence affects the increase in stress and strain intensity. Within the region of tunica albuginea adjacent to the plague, the increase factor of Von Mises stress was 3; in the plague, it was more than 5. The high stress intensity can be attributed to the pain symptoms of Peyronie's disease. The high local stress intensity is caused by the significant stiffness difference between the tunica albuginea and the plague. The material parameters in this study were based on literature data, which are limited in general. The material properties of the tunica albuginea and corpus cavernosa were adjusted to reflect the clinical observations and the chosen modeling strategy.

The results can be applied for the treatment of Peyronie's condition in which the rigidity of the plague is reduced by shock pulses. The effect of changes in mechanical parameters of the plague induced by the treatment can be rationally investigated using numerical simulations.

The numerical simulation presented in this report has a potential application in the diagnosis of Peyronie's disease and similar disorders. The numerical model can reflect in detail the anatomy of the tissue structure with malformations. The graphical visualization can improve understanding and communication with patients. The process is not invasive and well suited for analysis in the diagnosis phase. Parametric studies can be made to identify the effects of plague size and location in specific situations.

## Figures and Tables

**Figure 1:** Geometry of the model cross-section.

**Figure 2:** Mesh discretization of the penis model.

**Figure 3:** Cases of plague locations in the study.

**Figure 4:** Deformed state of the penis in scale 1 : 1.

**Figure 5:** Von Mises stress distribution in tunica albuginea in normal condition. Case 0.

**Figure 6:** Von Mises stress distribution in tunica albuginea with plague. Case A.

**Figure 7:** Histogram of penis deviation from the clinical research of Drlik [8].

**Figure 8:** Angulation and rotation of penis at artificial erection before surgical correction (Drlik [8]).

**Figure 9:** State after resection by “lengthening” method before patch implantation (Drlik [8]).

**Table 1:** Material parameters.

Material	*E* (MPa)	Poison's ratio (-)
Tunica albuginea	12.0	0.4
Corpus cavernosa	10.0	0.0
Skin	0.5	0.4
Glans	10.0	0.4
Plague	320.0	0.2

**Table 2:** Summary of simulation results.

Case	Tip displacement (mm)			Deviation (degree)	Von Mises stress (MPa)
	Δ_*x*_	Δ_*y*_	Δ_*z*_		
0	0.0	0.0	32.3	0.0	10.0
A	0.0	42.6	24.8	40.2	30.0
B	-12.6	6.4	28.7	15.6	17.7
C	-12.6	-6.4	28.7	15.6	17.7
D	-9.3	-16.3	27.9	20.4	19.5

## Data Availability

The data on clinical studies on Peyronie's disease used to support the findings of this study are available from the first author upon request. Please contact: MUDr Pavel Drlík, Central Military Hospital in Prague, U Vojenské nemocnice 1200 Praha 6-Střešovice, 16200, Czech Republic, email: pavel.drlik@uvn.cz. Data on ATENA numerical models supporting the results of the presented study are available upon request from the corresponding author. Please contact: Ing. Vladimir Cervenka, PH.D., Cervenka Consulting s.r.o., Na Hrebenkach 55, 150 00, Praha 5, email: vladimir.cervenka@cervenka.cz.

## Additional Points

*Attestation of Investigator Independence/Accountability/First Publication*. The authors had full access to all study data, take full responsibility for the accuracy of the data analysis, and have authority over manuscript preparation and decisions to submit the manuscript for publication. The manuscript, including related data, figures, and tables, has not been previously published and is not under consideration elsewhere. *Code Availability.* The numerical simulation was performed with the code ATENA, which is owned by the second author.
